# The Impact of Study Setting on Clinical Characteristics in Older Chinese Adults with Subjective Cognitive Decline: Baseline Investigation of Convenience and Population-Based Samples

This article has been retracted.

**DOI:** 10.1155/2021/5538323

**Published:** 2021-06-04

**Authors:** Mingyan Zhao, Guanqun Chen, Taoran Li, Can Sheng, Yuxia Li, Ying Han

**Affiliations:** ^1^Department of Neurology, Xuanwu Hospital of Capital Medical University, Beijing, China 100053; ^2^Department of Neurology, Tangshan Gongren Hospital, Tangshan, China 063000; ^3^National Clinical Research Center for Geriatric Disease, Beijing, China 100053; ^4^School of Biomedical Engineering, Hainan University, Haikou, China 570228; ^5^Center of Alzheimer's Disease, Beijing Institute for Brain Disorders, Beijing, China 100053

## Abstract

**Background:**

Subjective cognitive decline (SCD) is the earliest symptom stage of Alzheimer's disease (AD). Previous studies have shown that the study setting is an important influence factor of SCD. However, the effect of this factor among a Chinese population with SCD is not clear. Here, we aim to compare the clinical characteristics of SCD between a convenience and a population-based sample in China.

**Methods:**

We included a convenience sample of 212 SCD subjects and a population-based sample of 110 SCD subjects. We performed univariate analysis to evaluate the between-group differences in sociodemographic characteristics, neuropsychological performance, psychiatric conditions, different cognitive domains, and the SCD-plus criteria. Multiple linear regression model was established, adjusted for sex, age, and education, and compared the neuropsychological performance between the groups.

**Results:**

The convenience sample had more years of education, a higher family history of dementia, and higher neuropsychological and anxiety depression score than the population-based sample. Using sex, age, education, group as the independent variables, and neuropsychological score as the dependent variable, multiple linear regression model was established; a statistically significant neuropsychological score difference (MoCA-B, AVLT-H-N4, AVLT-H-N5, AVLT-H-N7, AFT, and STT-B) was found between the two samples. In the SCD cognitive domains, the population-based sample had more complaints about declines in their language and planning domains. For SCD-plus criteria in memory domain, the convenience sample had more complaints, worry, and cognitive decline within the last 5 years, along with medical help-seeking.

**Conclusion:**

There were some different characteristics among SCD individuals between convenience samples and population-based samples in China.

## 1. Introduction

Dementia is a serious public health problem. In 2015, the World Alzheimer Report showed that approximately 47 million people have dementia, and this number is expected to increase to 131 million by 2050 [1]. However, there is currently no effective therapeutic agent for mild cognitive impairment (MCI) and Alzheimer's disease (AD) [2, 3]. Effective interventions to delay or prevent pathologic cognitive decline should be targeted at the earliest symptomatic stages of subjective cognitive decline (SCD) [4].

Cognitive decline was initially described in 1982 [5] and later was conceptualized as subjective cognitive impairment, subjective memory impairment, subjective memory decline, and so on [6]. Epidemiological studies have shown that cognitively normal elderly with SCD is more likely to develop MCI or AD dementia [7–12]. However, SCD is not consistently associated with future cognitive impairment [13–15]. This discrepancy may be related to different definitions and research methods. Settings of recruitment lead to differences in SCD, including sociodemographic characteristics, clinical manifestations, *apolipoprotein E (APOE) ɛ4* status, and biological markers [16–20]. Some studies have shown that cognitively normal volunteers recruited in the community or in memory clinics were younger, better educated, and had a higher rate of a family history of AD than population-based samples [16, 17]. Subjects from clinical cohort with more memory concerns tend to have more severe AD pathology and have shown a higher annual rate of conversion to MCI or dementia than their community counterparts [12, 21]. One study showed that the recruitment methods influenced the associated biomarkers and affective symptomatology [22]. These above studies showed that different research environments lead to different characteristics. However, there are no previous studies that compared samples of a population with SCD across different study settings in China.

The aim of our study was to compare the clinical features, neuropsychological performance, and the decline in different cognitive domains as well as the SCD-plus criteria between a convenience sample and a population-based sample of SCD subjects in China. We hypothesized that there are different characteristics among Chinese SCD individuals in different study settings.

## 2. Materials and Methods

### 2.1. Participants

The convenience sample is part of the Sino Longitudinal Study on Cognitive Decline (SILCODE) project, which is a longitudinal cohort study aiming to develop a model for the ultraearly diagnosis of AD. Participants are continuously recruited through public advertisements and referrals from physicians, memory clinics, or informants. After demographic, clinical, and laboratory screening, subjects meeting the inclusion criteria were selected. Neuropsychological assessments, imaging examinations, and laboratory examinations were completed at baseline and follow-up. For details of the implementation process, see the SILCODE study published in 2019 [23]. The study recruited 579 eligible baseline subjects from March 2017 to September 2018, and from these, we selected 212 subjects who were diagnosed with SCD (Figure 1).

Population-based samples were selected from an epidemiological survey conducted in ShunYi District in Beijing, China. The purpose of this study was to investigate the incidence and characteristics of SCD in a Chinese population. Shunyi District consists of 12 towns, 7 district offices, and 6 subdistricts, with a total of 426 villagers' committees and 85 subdistrict committees. At the end of 2015, the region had registered 80,000 permanent residents aged 60 to 80. Sixteen committees were selected by stratified cluster random sampling, and 4,505 people were selected by preliminary questionnaire screening. Ultimately, 2,689 people took part in the survey. After applying the inclusion and exclusion criteria, 814 residents completed the clinical and neuropsychological assessments between September and November 2016. Details of the design and data collection of the study have been published previously [24]. We selected 110 SCD subjects based on the study objectives and diagnostic criteria (Figure 1).

### 2.2. Subject Selection Criteria

The diagnostic criteria are based on a SCD diagnostic framework published by Frank Jessen in 2014 [25]. SCD is defined as a self-experienced persistent decline in cognitive capacity in comparison with a previously normal status, unrelated to an acute event. The patient has normal age-, gender-, and education-adjusted performance on standardized cognitive tests, and they do not meet the diagnostic criteria for MCI and AD. An MCI diagnosis conforms to the criteria proposed by Jak and Bondi: meeting any of the following three criteria: (1) two indexes of the same cognitive domains were damaged (>1.0 SD); (2) all 3 cognitive domains were impaired (>1.0 SD); or (3) the Functional Activities Questionnaire (FAQ) ≥ 9 [26]. A diagnosis of AD was based on the Diagnostic and Statistical Manual of Mental Disorders, fourth edition (DSM-IV) [27], and a CDR score ≥ 1.

The inclusion criteria include the following: Han ethnicity, 60–80 years old.

The exclusion criteria include the following: (1) other nervous system diseases that can lead to cognitive decline, such as cerebrovascular disease, Parkinson's disease, brain tumors, brain trauma, and epilepsy; (2) other systemic diseases that can cause cognitive decline: anemia, thyroid dysfunction, and metabolic encephalopathy; (3) a general anesthesia history, a history of poisoning with carbonic oxide, a psychiatric disease, a serious physical disease, substance use, visual and auditory disorders, and/or cannot complete the neuropsychological examination.

### 2.3. Neuropsychological and Clinical Assessment

The neuropsychological assessment includes (1) neuropsychiatric assessment: HAMA (Hamilton Anxiety) and HAMD (Hamilton Depression); (2) global cognition: MoCA-B (Montreal Cognitive Assessment-Basic) [28]; (3) memory: AVLT-H (Auditory Verbal Learning Test-Huashan version) [29]; (4) executive function: STT-B (Trail Making Test B) and STT-A (Trail Making Test A) [30]; (5) language: AFT (Animal Fluency Test) [31] and BNT (Boston Naming Test) [32]; (6) daily life ability: ADL (Activities of Daily Living) [33]; and (7) except for a vascular disease etiology: HIS (the Hachinski Ischemic Index) [34]. Sociodemographic characteristics, medical history, lifestyle (smoking and drinking history), personal history (marital status and profession), and SCD-questionnaire 9 were obtained with a questionnaire [35]. The epidemiological survey of ShunYi district did not include the STT-A and BNT but include some other substitute indexes, executive function: Clock-Drawing Test (CDT-30); language: Verbal Fluency Test (animals and fruits) [24, 36].

A semistructured interview was used to evaluate the details of SCD. The interview was administered face to face by trained physicians. Our assessment of subjective cognitive decline covered five different cognitive domains, including memory, language, planning, attention, and any other cognitive decline. For each domain, the physician asked the patient if they had noticed a deterioration in function, i.e., do you think your memory has become worse? If the participant answered this question with yes, the physician further questioned about the SCD-plus features, i.e., associated worry (“Does this worry you?”), onset (“How long ago did you start to notice the decline?”), the performance in comparison to peers (“Compared to other people of your age, would you say that your performance is worse?”), and medical help-seeking (“Have you ever been to a doctor for these problems?”) [37].

### 2.4. Statistical Analyses

All statistical analyses were performed with SPSS (version 17.0); *p* < 0.05 was considered to be statistically significant. For the quantitative data, the Kolmogorov-Smirnov test and a Q-Q plot were used to test for normality. The first model was univariable. Nonnormal distribution data (age, education, MoCA-B, AVLT-H-N4, AVLT-H-N5, AVLT-H-N7, AFT, HAMD, and HAMA) are described with the median and interquartile, and the Mann-Whitney *U* tests were used to compare the differences between groups. Normal distribution data (STT-B) are described with the mean ± standard deviation (SD), and *t* tests were used to compare the differences between groups. Categorical variables (sex, medical history, smoking, drinking, personal history, SCD-plus features, and SCD-I domains) are described as percentages; the chi-squared (*χ*^2^) test was employed to assess differences between groups. The second model was multivariable; multiple linear regression analyses was established, adjusted for sex, age, and education, and compared the differences between the study setting and the neuropsychological scales (MoCA-B, AVLT-H-N4, AVLT-H-N5, AVLT-H-N7, AFT, and STT-B).

## 3. Results

### 3.1. Sociodemographic, Clinical, and Neuropsychological Characteristics of the Groups

A total of 322 SCD cases were analysed. The convenience sample included 212 cases from the SILCODE, and the population-based sample included 110 cases from the epidemiological survey data of ShunYi district (Figure 1). Both groups were more likely to be female, and the convenience sample was younger than the population-based sample, but there were no group differences. Compared with the population-based sample, the convenience sample had more years of education (12 [10–15] versus 6 [4–9], *p* < 0.001) and a higher rate of a family history of dementia (49 [23.1%] versus 3 [2.7%], *p* < 0.001) (Table 1).

The neuropsychological assessment (MoCA-B, AVLT-H-N4, AVLT-H-N5, AVLT-H-N7, AFT, and STT-B) in the convenience sample was superior to that in the population-based samples (*p* < 0.001) (Table 1). Using sex, age, education, group as the independent variables, and neuropsychological score as the dependent variable, multiple linear regression model was established; there were still significant differences between the two groups (*p* < 0.001) (Table 2). The convenience sample had higher anxiety and depression scores (HAMD 3 [1-5.75] versus 1.5 [0-4], *p* = 0.002; HAMA 4 [2–6] versus 1 [0-4], *p* < 0.001). In the convenience sample, an *APOE* examination was performed in 209 of 212 SCD, and 50 (23.92%) subjects had *APOE ɛ4*. The population-based samples were not assessed for *APOE.* Because of the experimental design, some of the low-education subjects did not complete the STT. In the population-based sample, STT test was conducted by 41 subjects. (Table 1).

### 3.2. SCD Domains and SCD-Plus Characteristics of the Groups

The differences in the SCD domains and the SCD-plus characteristics are given in Table 3. Due to the inclusion criteria, the 322 included participants (100%) reported a memory decline. Compared with the convenience sample, more subjects complained of a decline in the language (46.4% versus 30.7%, *p* = 0.005) and planning domains (30% versus 15.1%, *p* = 0.002) in the population-based samples, and there was a statistically significant between-group difference. For memory, the convenience sample had more SCD patients reporting worries (62.7% versus 22.7%, *p* < 0.001), cognitive decline within the last 5 years (82.5% versus 65.5%, *p* = 0.001), and medical help-seeking (7.5% versus 0.9%, *p* = 0.012).

## 4. Discussion

In the study, we compared the demographic, neuropsychological, cognitive domains, and SCD-plus features between a convenience sample and a population-based sample. The main findings of our study are (1) the convenience sample had more years of education and higher neuropsychological score, and (2) the convenience sample was more consistent with the SCD-plus features.

The recruitment settings usually include population-based samples, community-based volunteer samples, clinical samples, convenience samples, and mixed samples. In the convenience samples and mixed samples, it is normal to find mixtures of two types, it is also normal to find mixtures of clinical characteristics. The differences among samples are mostly the initiative of seek medical help (self-selection bias) [38]. The convenience sample was partly community- and partly clinically based. The results suggest that the convenience sample had more years of education, a higher rate of a family history of dementia and higher neuropsychological score. The population-based sample had a greater proportion of decline in the nonmemory cognitive domains, and the convenience sample was more consistent with the SCD-plus features. There were different characteristics among SCD individuals between different study settings.

This is the first study to compare the characteristics of SCD between different recruitment settings of the Chinese population. In regard to the sociodemographic characteristics, a previous researcher showed that subjects from the Open House Initiative which can be considered partly medical help seeking and partly community-based were more likely to be women and had a higher educational level and a higher rate of a family history of dementia than those from the Memory Unit [39]. Some studies have found that cognitively healthy control volunteers recruited through community-based cohorts or memory clinics are younger, better educated, and more likely to have a family history of AD than population-based control samples [16, 17].

Our results are consistent with these studies. Our convenience sample was younger than the population-based samples, but there were no group differences. This may be related to the fact that we chose people 60–80 years old. The convenience sample had a significantly higher rate of a family history of dementia. One possible explanation for this is a worry associated with a family history of dementia triggered medical help-seeking [18]. It is possible that highly educated individuals are more sensitive to subtle declines in cognitive function and pay more attention to cognition declines, leading to more help-seeking, so the convenience sample is better educated than the population-based samples. This may also be related to the fact that the target population of the convenience samples is biased depending on the channel of recruitment. In the convenience sample, most participants are highly educated individuals which are recruited through public advertisements and referrals. In the population sample, as the result of the stratification, we selected 2 subdistrict areas, 3 regional offices, and 4 towns; the sample represents the education of the general population. The convenience sample also had a lower proportion of hypertension, a higher proportion of dyslipidemia, and a lower proportion employed in physical labor. Their effects on cognitive decline are inconclusive.

SCD subjects compared to controls had lower scores on neuropsychological performance but within the normal range, which is predictive of a future decline [7]. A previous study showed different neuropsychological characteristics depending on the recruitment method. The Open House Initiative sample showed better overall neuropsychological performance than the Memory Unit sample on global cognition, two executive tasks, and on recognition memory [39]. It has been demonstrated that memory clinic patients with MCI have poorer cognitive performance and a higher risk of progression to dementia than population-based samples [17]. Our results are different from previous studies in this regard. It may be related to the difference in educational level between these two groups. Although we adjusted for education, the underlying pathological basis may still influence the results. In less-educated individuals, a degree of underlying brain pathology might lead to clinical symptoms. Highly educated individuals may be able to compensate for longer periods of time and appear clinically normal because of a higher cognitive reserve. Cognitive reserve has the potential to delay or slow cognitive decline in individuals with SCD [40]. SCD individuals with more years of education have a stronger amyloid burden compared with less-educated individuals. The association between SCD and A*β* burden becomes stronger in greater educational individuals [41].

Most psychiatric disorders and subclinical psychiatric conditions can affect cognition. Recruitment methods influence the affective symptomatology. Depression, for example, is specifically associated with medical help-seeking. There are higher rates of depression/anxiety symptomatology in clinical-based SCD samples compared with community-based SCD samples [18, 42]. Despite not meeting the criteria for a clinical diagnosis of depression, a cross-sectional study showed that subclinical depression was more prevalent in medical-help seeking SCD individuals compared to community-recruited older adults [22]. In our study, people with significant anxiety and depression were excluded, but the anxiety and depression scores of the convenience sample were significantly higher than the population-based samples. This is because the convenience samples are seeking medical help more actively.

Several community-based studies have revealed that the rate of cognitive complaints is relatively high in the typical older adult population and could represent complaints about normal aging [43–45]. This may result in false-positive diagnoses of SCD. In memory clinics, cognitive complaints are more likely to reflect nonnormal aging, which eliminates false-positives [46]. Thus, the evaluation of the SCD concept in preclinical AD population remains to be further explored. In 2014, the SCD-Initiative proposed the “SCD-plus criteria” as an enrichment strategy for the likelihood of preclinical AD in individuals with SCD [25]. In addition, current research suggests the SCD assessments should involve additional cognitive domains [47].

In our study, we used a semistructured interview to assess SCD features. The semistructured interview includes five different cognitive domains (memory, language, planning, attention, and any other cognitive decline) and comprises all five SCD-plus features. Due to the inclusion criteria, all SCD patients reported a decline in memory. In the other domains, language complaints were the most frequent, followed by an attention, planning, and any other cognitive decline. A recent study showed the prevalence for SCD of affected different cognitive domains was language (82.9%), planning (21%), attention (46.7%), and any other cognitive decline (37.1%) [37]. The use of different inclusion criteria and research methods can lead to a different result. One study showed word finding difficulties accounted for three-quarters of SCD individuals, which reflect its association with a better cognitive performance [37]. The incidence is similar in MCI and community cognitively healthy older adults, suggesting that subjective word finding difficulty is a part of normal aging rather than a possible sign of AD pathology [48]. In our study, the population-based samples had more subjective complaints of declines in the language domain than did the convenience sample. The decline of cognitive domains in the population-based samples has greater consistency with normal aging. This supports the potential of convenience samples to have greater consistency with preclinical SCD.

The two participant groups differed in their decline of SCD-plus features. Longitudinal and cross-sectional studies acknowledge complaints of memory changes are nonspecific, unless associated with a progressive nature or worry [49, 50]. In our study, the proportion of SCD individuals with worry in the convenience sample is much higher than that in the population-based sample. A study reported 81% SCD participants reported the onset of their decline within the last 5 years. This is based on direct testing, and it validated the SCD-plus criterion “onset within the last 5 years” was significantly associated with amyloid pathology [37]. The reported onset within the last 5 years in the SCIENCE SCD-cohort was 83% [51]. These findings are completely consistent with the reported onset in our study, where 82.5% reported an onset within the last 5 years in the convenience sample. Memory changes and a worse memory in comparison to peers are useful for identifying individuals at preclinical and prodromal stages of AD [52]. In our study, the proportion of SCD participants reported they had a worse memory in comparison to peers was 27.8% in the convenience sample and 24.5% in the population-based samples. The former is closer to the previous results of 29.5% [37]. It has been reported that medical help-seeking groups have more pronounced markers of neurodegeneration at a higher prevalence than healthy community-dwelling volunteers [22, 50]. The above research confirmed that the convenience sample is more closely associated with SCD-plus features than the population-based samples.

Our study of cognitive domains and SCD-plus features indicated that the population-based samples are more consistent with normal aging, and the convenience sample is more closely associated with SCD-plus features. But the population-based samples performed significantly worse in neuropsychological performance compared to the convenience samples. It may be related to the fact that different levels of education result in neuropsychological performance and underlying pathological basis. This may also be related to the fact that the target population of the convenience samples are biased depending on the channel of recruitment. We should consider the representativeness of the samples in future SCD studies. Longitudinal studies of different samples are necessary; SCD-plus features or worse neuropsychological performance is better predictors of future cognitive decline in certain samples. We acknowledge that there are some limitations of this study. First, this is a retrospective study, and some details of the two samples were not identical, but the principles of diagnosis are consistent. Second, there were no genetic or imaging data available for the population-based samples, so we cannot compare their biomarkers of AD. We will perform a follow-up of this cohort in the future.

## 5. Conclusions

There are differences in demographic, neuropsychological, cognitive domains and SCD-plus features among SCD subjects from different recruitment settings in China. The convenience sample was more consistent with SCD-plus features than the population-based sample. Thus, the impact of study setting on SCD individuals also needs to be considered in the future. Study setting is an essential factor result in the heterogeneity of SCD. When choosing the subjects or analyzing research results, the role of study setting should be taken into account.

## Figures and Tables

**Figure 1:** The flow charts of this study. NC: normal controls; SCD: subjective cognitive decline; MCI: mild cognitive impairment; AD: Alzheimer's disease.

**Table 1:** Demographics and neuropsychological assessments.

	Convenience sample (*n* = 212)	Population sample (*n* = 110)	*χ* ^2^/*t*/*Z*	*p*
Age, y	65 (63-69)	67 (63-70)	-1.940	0.052^d^
Female, *n* (%)	140 (66%)	74 (67.3%)	0.050	0.824^c^
Education, y	12 (10-15)	6 (4-9)	-12.801	<0.001^d^
MoCA-B	26 (24-27)	20 (17-22)	-12.484	<0.001^d^
AVLT-H-N4	7 (6-9)	4 (3-5)	-11.787	<0.001^d^
AVLT-H-N5	7 (5.25-8)	3 (2-4)	-12.276	<0.001^d^
AVLT-H-N7	23 (22-24)	20 (19-22)	-8.438	<0.001^d^
AFT	19 (16-22)	13 (11-16)	-9.758	<0.001^d^
STT-B^b^	135.85 ± 33.77	176.24 ± 41.33	-6.749	<0.001^e^
HAMD	3 (1-5.75)	1.5 (0-4)	-3.100	0.002^d^
HAMA	4 (2-6)	1 (0-4)	-6.647	<0.001^d^
*APOEε4* ^a^	50 (23.92%)	—		
Hypertension, *n* (%)	79 (37.3%)	57 (51.8%)	6.288	0.012^c^
Diabetes, *n* (%)	29 (13.7%)	12 (10.9%)	0.500	0.479^c^
Dyslipidemia, *n* (%)	78 (37%)	27 (24.5%)	5.068	0.024^c^
Smoking, *n* (%)	46 (21.7%)	26 (23.6%)	0.157	0.692^c^
Drinking, *n* (%)	50 (23.6%)	27 (24.5%)	0.037	0.848^c^
Married, *n* (%)	181 (85.4%)	96 (87.3%)	0.216	0.642^c^
Job category, *n* (%)				
Mental	148 (69.8%)	11 (10%)	150.082	<0.001^c^
Physical	30 (14.2%)	92 (83.6%)		
Mental+physical	34 (16%)	7 (6.4%)		
Family history	49 (23.1%)	3 (2.7%)	22.227	<0.001^c^

All continuous variables in the table were nonnormally distributed and described as median (interquartile). ^a^APOE genotype results were included in the convenience sample SCD subjects (*N* = 209), *ε*4^+^ (*N* = 50). ^b^STT-B results were included in the convenience sample (*N* = 212) and in population-based samples (*N* = 41). ^c^The *p* value was calculated using Chi-square. ^d^The *p* value was calculated using the Mann-Whitney *U*. ^e^The *p* value was calculated using independent samples *t* tests. MoCA-B: Montreal Cognitive Assessment-Basic; AVLT-H-N4: Auditory Verbal Learning Test-Huashan version short-delayed free recall (5 min); AVLT-H-N5: Auditory Verbal Learning Test-Huashan version long-delayed free recall (20 min); AVLT-H-N7: Auditory Verbal Learning Test-Huashan version long-delayed recognition (20 min); AFT: Verbal Fluency Test (animal); STT-B: Shape Trail Test B; HAMD: Hamilton Depression Rating Scale; HAMA: Hamilton Anxiety Scale.

**Table 2:** Multivariable compared the neuropsychological assessments.

	*B* (*95%CI)*	*t*	*P*
MoCA-B	-3.662 (-4.483, -2.842)	-8.782	<0.001
AVLT-H-N4	-2.605 (-3.238, -1.972)	-8.093	<0.001
AVLT-H-N5	-2.719 (-3.359, -2.079)	-8.359	<0.001
AVLT-H-N7	-1.633 (-2.204, -1.061)	-5.622	<0.001
AFT	-2.995 (-4.334, -1.656)	-4.401	<0.001
STT-B	32.143 (20.035, 44.250)	5.229	<0.001

MoCA-B: Montreal Cognitive Assessment-Basic; AVLT-H-N4: Auditory Verbal Learning Test-Huashan version short-delayed free recall (5 min); AVLT-H-N5: Auditory Verbal Learning Test-Huashan version long-delayed free recall (20 min); AVLT-H-N7: Auditory Verbal Learning Test-Huashan version long-delayed recognition (20 min); AFT: Verbal Fluency Test (animal); STT-B: Shape Trail Test B.

**Table 3:** SCD-plus features and SCD-I domains.

	Convenience sample (*n* = 212)	Population sample (*n* = 110)	*χ* ^2^	*p*
Decline in memory	212 (100%)	110 (100%)		
Particular concerns/worries	133 (62.7%)	25 (22.7%)	46.386	<0.001
Onset within 5 years	175 (82.5%)	72 (65.5%)	11.843	0.001
Feeling worse than peers	59 (27.8%)	27 (24.5%)	0.399	0.528
Medical help-seeking	16 (7.5%)	1 (0.9%)	6.381	0.012
Decline in language	65 (30.7%)	51 (46.4%)	7.749	0.005
Particular concerns/worries	35 (53.8%)	15 (29.4%)	6.957	0.008
Onset within 5 years	56 (86.2%)	36 (70.6%)	4.220	0.040
Feeling worse than peers	19 (29.2%)	20 (39.2%)	1.277	0.259
Medical help-seeking	1 (1.5%)	0 (0%)		1.000^∗^
Decline in planning	32 (15.1%)	33 (30%)	9.987	0.002
Particular concerns/worries	14 (43.8%)	10 (30.3%)	1.261	0.261
Onset within 5 years	28 (87.5%)	21 (63.6%)	4.986	0.026
Feeling worse than peers	4 (12.5%)	15 (45.5%)	8.529	0.003
Medical help-seeking	1 (3.1%)	0 (0%)		0.492^∗^
Decline in attention	66 (31.1%)	30 (27.3%)	0.516	0.473
Particular concerns/worries	34 (51.5%)	11 (36.7%)	1.826	0.177
Onset within 5 years	55 (83.3%)	20 (66.7%)	3.352	0.067
Feeling worse than peers	12 (18.2%)	10 (33.3%)	2.680	0.102
Medical help-seeking	2 (3%)	0 (0%)		1.000^∗^
Decline in other	13 (6.1%)	1 (0.9%)		0.059^∗^

^∗^The *p* value was calculated using Fisher's Exact Test.

## Data Availability

The data used to support the findings of this study are available from the corresponding author upon request.
